The article "Characterization of recombinant fructose-1,6-bisphosphatase gene mutations: evidence of inhibition/activation of FBPase protein by gene mutation" was published in 2019. Journal: Biosci Rep.

# Characterization of recombinant fructose-1,6-bisphosphatase gene mutations: evidence of inhibition/activation of FBPase protein by gene mutation

**DOI:** 10.1042/BSR20180960

**Published:** 2019-02-22

**Authors:** Gemma Topaz, Victor Epiter-Smith, Cristina Robalo, Megan Emad, Vanessa Ford, Jadine Daley, Jennifer Byron, Kimberly A. Stieglitz

**Affiliations:** 1 Boston University, Biology Department, Boston, MA, U.S.A.; 2 Roxbury Community College, STEM Biotechnolgy Division, Roxbury, MA, U.S.A.

**Keywords:** allosteric regulation, enzymatic activity, hyperglycemia, hypoglycemia, mutagenesis

## Abstract

Specific residues of the highly regulated fructose-1,6-bisphosphatase (FBPase) enzyme serve as important contributors to the catalytic activity of the enzyme. Previous clinical studies exploring the genetic basis of hypoglycemia revealed two significant mutations in the coding region of the FBPase gene in patients with hypoglycemia, linking the AMP-binding site to the active site of the enzyme. In the present study, a full kinetic analysis of similar mutants was performed. Kinetic results of mutants Y164A and M177A revealed an approximate two to three-fold decrease in inhibitory constants (*K*_i_’s) for natural inhibitors AMP and fructose-2,6-bisphosphate (F2,6-BP) compared with the Wild-type enzyme (WT). A separate mutation (M248D) was performed in the active site of the enzyme to investigate whether the enzyme could be activated. This mutant displayed an approximate seven-fold increase in *K*_i_ for F2,6-BP. Interfacial mutants L56A and L73A exhibited an increase in *K*_i_ for F2,6-BP by approximately five-fold. Mutations in the AMP-binding site (K112A and Y113A) demonstrated an eight to nine-fold decrease in AMP inhibition. Additionally, mutant M248D displayed a four-fold decrease in its apparent Michelis constant (*K*_m_), and a six-fold increase in catalytic efficiency (CE). The importance—and medical relevance—of specific residues for FBPase structural/functional relationships in both the catalytic site and AMP-binding site is discussed.

## Introduction

Fructose-1,6-bisphosphatase (FBPase) is a complex tetramer and a highly regulated enzyme. FBPase activity is regulated synergistically by the allosteric inhibitors AMP and fructose-2,6-bisphosphate (F2,6-BP). As an enzyme, FBPase functions in the degradation of fructose-1,6-bisphosphate (FBP), which hydrolyzes to fructose-6-phosphate (F6P) and inorganic phosphate [1]. FBPase is a key rate-controlling enzyme in the gluconeogenic pathway. Individuals with FBPase deficiency exhibit hypoglycemia and metabolic acidosis due to impaired gluconeogenesis. In rare cases, hypoglycemia, an autosomal recessive disorder characterized by insufficient blood glucose levels, has been genetically linked to FBPase deficiency in clinical studies [2]. Since hypoglycemia has been found associated with FBPase mutations, impaired or mutated FBPase has proven to be a contributor to hypoglycemia [2]. It is plausible that a genetic link may also exist between hyperglycemia and FBPase mutations.

The article "Characterization of recombinant fructose-1,6-bisphosphatase gene mutations: evidence of inhibition/activation of FBPase protein by gene mutation" was published in 2019. Journal: Biosci Rep.

Hyperglycemia, defined by an excess of glucose in the bloodstream, is most commonly associated with Type II Diabetes, characterized by chronic elevations of plasma glucose concentrations. Hyperglycemia affects nearly 29 million people in the United States alone, and results from a relative deficiency of insulin action [3–5,8]. Additional medical conditions associated with diabetes include retinopathy, neuropathy, increased risk of cardiovascular disease, and stroke [6–9]. In the present study, mutations in the target enzyme (mammalian FBPase) were designed to better define the role of specific residues involved in the regulation of FBPase, and to characterize the catalytic variations of mutated FBPase. The AMP-binding site mutants were selected based on a previous study of the 3D structure of FBPase complexed to AMP in which a hydrogen bonding network from the AMP-binding site to the active site of the enzyme was identified [10]. Several amino acids mutated in this study may also play a critical role in transmitting the allosteric signaling from the AMP site to the active site of the enzyme, as they link the AMP-binding site to the active site of FBPase. In addition, results from previous studies confirm that a genetic basis for hypoglycemia exists in the coding region of the FBPase enzyme, also strongly suggesting that a genetic basis for hyperglycemia may exist as well [2]. As a follow-up to the observations of previous studies *in vivo* and this study *in vitro*, a genetic basis for hyperglycemia may be confirmed in the clinical setting, and the presence of an additional pathological link to Type II Diabetes would then be established. Findings from future clinical studies could provide further motivation for the investigation and design of more potent and bioavailable inhibitors against FBPase [11–13].

## Materials and methods

### Design of pig kidney FBPase mutants/site-directed mutagenesis

To determine if specific mutations cause disruption in enzymatic activity and structural changes, site-directed mutagenesis was done on selected residues. Site-directed mutagenesis was performed using seven different pig kidney FBPase primer sequences via PCR, amplifying single strands or plasmids of interest [14,15]. The pig kidney FBPase gene was readily available from American Type Culture Collection (ATCC). All other chemicals and materials for the present study were purchased from VWR or Sigma–Aldrich chemical company. The construct was made with the pig kidney FBPase and modeled after the lac operon expression system with ampicillin resistance. The construct was utilized to overexpress and purify a mammalian FBPase enzyme (pig kidney FBPase) with higher solubility than the human gene product (cleavage of histidine tag after column chromatography in human FBPase caused low solubility). The subcloning procedure and plasmid modification for histidine 6mer C-terminus tail for purification via Nickel NTA Affinity Column was performed as previously described [1]. The first two constructed mutant pig kidney FBPase plasmid DNA were mutated from 490_G_to_A (amino acid coding from tyrosine to alanine–Y164A) and 530_G_to_A (coding from methionine to alanine–M177A). Both were used to confirm, and to correlate with, clinical data on site-directed mutagenesis and kinetics on purified mutant FBPase protein. Lysine to alanine (K112A) and tyrosine to alanine (Y113A) mutant plasmids were used as models based on results from previous studies of mutations of lysine to glutamine (K112Q) and tyrosine to phenylalanine (Y113F) enzymes, respectively [16]. At last, new mutant plasmids were designed for mutant protein M248D (Met^248^), L56A (Leu^56^), and L73 (Leu^73^), which were done via visual inspection of the active site and areas near tetramer interface (where PFE ({4-[3-(6,7-diethoxy-quinazolin-4-ylamino)-phenyl]-thiazol-2-yl}-methanol) binds; Figure 2A) in the graphics program Chimera to investigate if activity could be enhanced/altered as a result of mutation [17].

The article "Characterization of recombinant fructose-1,6-bisphosphatase gene mutations: evidence of inhibition/activation of FBPase protein by gene mutation" was published in 2019. Journal: Biosci Rep.

### Transformation(s) and purification of mutant plasmids

In order to overexpress, isolate, and purify recombinant mutant enzymes, transformations and purification of mutant plasmids was performed. Following site-directed mutagenesis, each of the mutant plasmids underwent transformation with XL Blue super-competent cells [18,19]. Cells were plated on LB agar plates and colonies were selected for 5 ml overnight for plasmid purification using various kits [20,21]. Following purification, mutant plasmids were screened for integrity as they were run on an agarose gel and sequenced. Cell colonies were selected then grown overnight in 5 ml LB AMP broth. Colonies were scaled up between 1 and 2 l and protein samples were then isolated and purified.

A transformation for overexpression was then performed as previously described [22], and a preheated water bath was established at 42°C. BL21 (DE3) competent *Escherichia coli* cells were removed after being frozen at −80°C and thawed on ice. A 50-µl volume of competent cells was added to an empty Eppendorf tube with 2.0 µl of plasmid (1–20 ng plasmid DNA) [22], and the tubes were cooled on ice for 30 min. Tubes containing bacteria were then subjected to heat shock using a 42°C water bath for 45 s, before being transferred and incubated on ice for 15 min. A volume of 400 µl of sterile LB broth was added. The tube was then placed into a roller drum at 37°C at 20 rpm for 60 min, followed by centrifugation in a tabletop microcentrifuge at 3000 rpm for 5 min. The leftover supernatant was then discarded; 450 µl of sterile LB broth was added and clumping cells were pipetted and re-suspended. The contents of the tubes were transferred to LB Ampicillin plates using sterile technique. Plates were then incubated for 18 h at 37°C and stored for 2.5 weeks at 4°C.

The article "Characterization of recombinant fructose-1,6-bisphosphatase gene mutations: evidence of inhibition/activation of FBPase protein by gene mutation" was published in 2019. Journal: Biosci Rep.

### Protein overexpression, isolation, and purification

To prepare the recombinant WT and mutant enzymes for kinetic and binding assays, the recombinant proteins were overexpressed, isolated, and purified. Single colonies were selected and 5 ml cultures were grown overnight. The culture medium was shaken overnight at a temperature of 37°C. The following day, 1 l LB AMP medium was inoculated with the 5 ml cultures overnight and incubated at 37°C for 2–3 h. Host cell health and growth was measured using a spectrophotometer at optical density (OD) 580 nm assessing cell density. Once the OD was between 0.4 and 0.6, indicating optimal density for overexpression as previously determined, the culture was inoculated with 1 ml of 1000× IPTG (0.8 Molar in water) as described previously [21]. The host cell translation was inhibited with 34 mg/ml chloramphenicol (in isopropanol) [23]. The solution was shaken again for 2–3 h at 37°C to ensure optimal growth of the host cells.

Cells were then isolated by pelleting in 250 ml flasks in a centrifuge at 4000 rpm. After the cells were frozen, each cell pellet was re-suspended in 20 ml of 50 mM Tris pH 7.5. The supernatant underwent lysis via sonication to release cell contents. Each protein solution was sonicated as previously described [23]. Sonication setting was at 10% duty cycle for 5 min, pulsing 10 s on and 10 s off ×3. Each supernatant cell lysate was centrifuged for 30 min at 13500 rpm at 4°C and transferred to dialysis tubing for dialysis in 50 mM Tris pH 8.0. Each protein was then purified via NTA nickel affinity column as previously described [24].

Briefly, buffer with low imidazole (50 mM) in 50 mM Tris pH 7.5 was washed through an NTA nickel affinity column after loading WT or mutant protein in 50 mM Tris pH 7.5. This initial wash in low imidazole buffer was performed in order to elute proteins containing histidine from host bacteria. The recombinant WT and mutant enzymes were eluted from the NTA nickel affinity column in 300 mM imidazole, 50 mM Tris buffer pH 7.5. In addition, gel filtration was run on a G250 column in Tris buffer pH 7.5 in 0.150 M NaCl as eluent buffer to investigate the oligomeric status of mutants compared with WT enzyme.

The article "Characterization of recombinant fructose-1,6-bisphosphatase gene mutations: evidence of inhibition/activation of FBPase protein by gene mutation" was published in 2019. Journal: Biosci Rep.

### Characterization of purified mutant enzymes and preparation for enzyme kinetic assays

The purity of the recombinant WT and mutant enzymes was assessed via SDS/PAGE, and the oligomeric state was identified with native gel electrophoresis. An SDS/PAGE gel electrophoresis was used to separate and identify proteins with the correct molecular weight [25]. Figure 1 shows both SDS and native gels for WT and mutant enzymes. The 12% polyacrylamide gel for Figure 1A was made in Tris buffer with 2% SDS. The sample buffer was 100 mM Tris pH 6.8, 2% SDS, 5% β-mercaptoethanol, and 15% glycerol. Figure 1A shows the purified WT as well as each mutant. The oligomeric state of each mutant was also investigated by running a native Tris gel (polyacrylamide gel without SDS, and sample buffer without SDS and β-mercaptoethanol) after gel filtration for both WT and each mutant (Figure 1B).

**Figure 1:** Analysis of enzyme purity and oligomer enzyme structure using gel electrophoresis (**A**) **SDS/PAGE of purified WT and mutants.** Purity of WT and mutant enzymes after His-Tag purification scheme was assessed prior to kinetic/binding assays using 12% SDS/PAGE gel electrophoresis. Viewing from left to right, standard molecular weight markers, WT and mutant enzymes: Y164A, M177A, L56A, L73A, K112A, Y113A, and M248D. Purified enzymes were loaded on to gel with concentrations ranging from 2.5 to 5.0 µg/µl. (**B**) **Native (TRIS) gel analysis of WT and mutants.** Oligomeric state of WT and mutant enzymes was assessed using 12% polyacrylamide native TRIS gel. Viewing from left to right, WT and mutant enzymes: Y164A, M177A, L56A, molecular weight markers, L73A, K112A, Y113A, M248D. Purified enzymes were loaded on to native gel after gel filtration and concentrating each enzyme to 50×.

For the kinetic assay, a standard curve was obtained from an ammonium molybdate Malachite Green inorganic phosphate assay (OD660 nm) [25]. The purified FBPase protein was dialyzed ×3 in 50 mM Tris buffer at pH 7.5 at 4°C. For enzyme concentration, absorbency values were recorded for all five mutant proteins using spectrophotometer readings at OD280 nm. To quantitate enzyme concentration, the enzymes were calculated based on the quantity of micrograms per microliter (µg/µl) present. Final concentration of WT and mutant enzymes was between 2.5 and 5.0 µg/µl. Using a colorimetric assay as described below, specific activity (SA) was determined. At last, all kinetic and binding assays described below were performed in 50 mM Tris pH 7.5.

The article "Characterization of recombinant fructose-1,6-bisphosphatase gene mutations: evidence of inhibition/activation of FBPase protein by gene mutation" was published in 2019. Journal: Biosci Rep.

### Kinetic assays on mutant enzymes

Kinetic assays were performed for WT and mutant enzymes to identify functional differences between the WT enzyme and the mutants. A Malachite Green colorimetric assay based on the complex formed between Malachite Green, ammonium molybdate, and the product of inorganic phosphate cleaved from the substrate FBP under acidic conditions, was used with varying substrate FBP concentrations (100–500 µM) [21,22,26] in 50 mM Tris buffer pH 7.5 at 37°C with 5 mM MgCl_2_. Readings recorded at OD660 nm for each enzyme were applied to the standard curve equation. Micromoles of inorganic phosphate were calculated to determine the SA of mutant enzymes.

For each clone, the kinetic assay was performed in duplicates of triplicates. Malachite Geen was used to detect inorganic phosphate. Two separate clones were processed independently of the same mutant. All kinetic data were fit to symmetric sigmoidal curve using Origin software based on methods previously described [27–29]. More specifically, for kinetic parameters established via curve fitting (shown in Tables 1–3; and in Figure 5A,B), the equation y = d + (a − d)/1 + (x/c)^b^ was used where ‘x’ is represented by apparent Michelis constant (*K*_m_) when y = *V*_max_. The association (binding) constant (*K*_a_) value for magnesium as well as the Hill coefficient for AMP and magnesium metal were obtained via saturation curves, fitting the data to the Hill equation as previously described [28,29]. *P*-values were significant at <0.001 and represent a comparison with the WT enzyme.

**Table 1:** Kinetic data of pig kidney FBPase AMP and F2,6-bisphosphate sensitivity comparing mutants and WT*

Enzyme	IC_50_ (µM)		IC_50_ change (mutant/WT)	
	AMP	F2,6-BP	AMP	F2,6-BP
K112A_1	68.5 (± 1.36)	1.50 (± 0.05)	9.10	1.00
K112A_2	52.3 (± 1.04)	1.50 (± 0.04)	7.00	1.00
Y113A_1	48.6 (± 0.97)	1.80 (± 0.03)	6.50	1.20
Y113A_2	55.3 (± 1.10)	1.70 (± 0.06)	7.40	1.10
Y164A	2.50 (± 0.08)	0.95 (± 0.08)	0.33	0.63
M177A_1	3.50 (± 0.05)	0.75 (± 0.06)	0.47	0.50
M177A_2	3.90 (± 0.06)	0.62 (± 0.07)	0.52	0.41
L56A	7.35 (± 0.09)	7.50 (± 0.15)	0.98	5.00
L73A	6.95 (± 0.08)	7.25 (± 0.14)	0.93	4.83
M248D	7.20 (± 0.30)	10.5 (± 0.12)	0.96	7.00
WT	7.50 (± 0.30)	1.50 (± 0.03)	N/A	N/A

* Concentration of FBP substrate tested for AMP and F2,6-BP IC_50_ varied from 10 to 50 µM. Assays were performed in triplicates and averaged. AMP inhibitor was tested from 2.5 to 80 µM and F2,6-BP inhibitor from 2.5 to 50 µM.

### Differential scanning fluorimetry assay

Differential scanning fluorimetry (DSF) assays were designed and implemented to run on WT and each mutant for the purpose of determining relative stabilities by melting point, and to detect structural changes in the enzymes upon ligand binding. Thermal shift assays were performed with a Light Cycler 96 System Real-Time PCR machine (Roche) using Sypro-Orange dye (Invitrogen) and thermal ramping (0.25°C per min between 20 and 85°C). All proteins were diluted to 5 µM in 50 mM Tris pH 7.5 and 150 mM NaCl in the presence and absence of either AMP inhibitor or cofactor magnesium. Neither FBP substrate nor F2,6-BP inhibitor could be assayed due to fact that they both began decomposing at and above approximately 50°C. Data were processed using the Boltzmann equation to generate sigmoidal denaturation curves, and average *T*_m_/Δ*T*_m_ values were calculated as previously described using GraphPad Prism software package [30].

The article "Characterization of recombinant fructose-1,6-bisphosphatase gene mutations: evidence of inhibition/activation of FBPase protein by gene mutation" was published in 2019. Journal: Biosci Rep.

## Results

### Demonstration of the purity and identity of oligomeric state of WT and mutant enzymes

Figure 1 shows both SDS and native gels for WT and mutant enzymes. The purified WT monomer as well as each mutant monomer is presented in Figure 1A, and the oligomeric state of each mutant and WT is shown in Figure 1B.

Figure 1A confirms that the WT and mutant enzymes were purified to a similar level of purity before use in the subsequent kinetic and binding assays. Moreover, a native gel of the WT and mutant enzymes (shown in Figure 1B) following gel filtration revealed that all of the mutant enzymes had tetrameric states.

### Sequence comparison of human and pig kidney enzymes

Although the pig kidney FBPase was used to perform these mutations, all of the mutated residues have shown to align with the human FBPase. As depicted by the sequence alignment in Figure 2, there is high homology between the pig kidney and human FBPase.

**Figure 2:** Complimentary amino acid sequence alignment comparison of the human and pig kidney FBPases

The gaps in the alignment are indicated by dashed lines. A dot is indicated at every ten identical residues are indicated by asterisks. Top sequence is human FBPase the bottom sequence is pig kidney FBPase.

Amino acid sequences for pig and human liver show >90% identity (Figure 2). Coding differences are indicated by dashed lines. Importantly, the active site residues in addition to residues found mutated in clinical studies—as well as other residues mutated in the present study—are identical for human and pig kidney. It is therefore a reasonable substitution to utilize the more soluble purified recombinant pig kidney FBPase than the less soluble human enzyme.

### Structural analysis of pig kidney FBPase

Figure 3A presents a structural overlay for both human and pig kidney FBPases, illustrating that both are tetramers which share nearly identical tertiary structure (pig kidney tetramer PDB code: 1KZ8, human tetramer PDB code: 1FTA) [31,32]. Furthermore, the three regions responsible for the regulation of this enzyme are indicated in Figure 3A as: (i) the AMP-binding site: the site of natural negative allosteric regulation; (ii) the active site: the site of homotropic allosteric regulation by means of the F2,6-bisphosphate inhibitor; and (iii) the novel PFE tetramer-binding site: a second site for negative allosteric regulation [31]. Mutations were strategically selected in each of these three regions as well as the interface between the sites, to study their kinetic effects.

The article "Characterization of recombinant fructose-1,6-bisphosphatase gene mutations: evidence of inhibition/activation of FBPase protein by gene mutation" was published in 2019. Journal: Biosci Rep.

**Figure 3:** Structural overlays of tetramer human FBPase (PDB code: 1FTA [32]) with pig kidney FBPase (PDB code: 1KZ8 [31]): identification of strategically positioned residues selected for mutation (**A**) **The three distinct regions of the enzyme.** 1) The AMP-binding site; 2) The active site; and 3) A novel PFE allosteric inhibitor-binding site [31]. Blue structure is pig kidney 1KZ8 and tan structure is human 1FTA. (**B**) **Structural overlay showing the strategic position of residues L73 and L56 (shown in magenta).** The active site cavity is shown on the left, and the PFE allosteric binding site is shown on the right of the two residues. Blue structure is pig kidney 1KZ8 and tan structure is human 1FTA. (**C**) **Structural overlay showing the location of M177 and Y164 residues (shown in magenta)**. The residues are shown strategically positioned between the two active sites of the dimer and the AMP-binding site. Blue structure is pig kidney1KZ8 and tan structure is human 1FTA. (**D**) **Structural overlay showing the position of Y113 and K112 residues (shown in magenta).** These AMP-binding site residues are shown in close proximity to residues M177 and Y164. Blue structure is pig kidney 1KZ8 and tan structure is human 1FTA. (**E**) **Structural overlay showing the position of residue M248 (shown in magenta).** The M248 residue is shown in close proximity to residues D121, E280, and D118, and activating metal manganese (shown in purple). Blue structure is pig kidney 1KZ8 and tan structure is human 1FTA.

As shown in Figure 3, the FBPase pig kidney tetramer overlay of human and pig kidney (PDB codes: 1FTA and 1KZ8) showed nearly identical orientation and conformation in the active site, AMP allosteric binding site, and PFE allosteric binding site architecture with an overall RMSD ∼1.8 Angstrom squared. In Figure 3B, the significance of the position between the two residues chosen for mutation is that L56 co-ordinates the PFE ligand, as does residue L73; both of which exhibit hydrophobic interactions with the ligand in the PFE-binding site. In addition, L73 and L56 are part of a network that leads from the allosteric binding site to the active site of the enzyme.

The article "Characterization of recombinant fructose-1,6-bisphosphatase gene mutations: evidence of inhibition/activation of FBPase protein by gene mutation" was published in 2019. Journal: Biosci Rep.

Other residues shown within the aforementioned network are V48 and L120. This hydrophobic network may stabilize previously described hydrogen bonding networks [10] including residues R49, S169, and D127, shown in the network, leading to the active site where the metal binds D121, D118, and E280. In Figure 3C, the M177 and Y164 interfacial residues are positioned between the AMP-binding site and active sites. Both of these residues have been found to be mutated in humans with hypoglycemia [2]. Note that the position of Y164 allows for the interaction and stabilization of the enzyme active site residue D121 in close proximity to M248, and via water, interacts with F6P oxygen atoms from hydroxyl functional groups (Figure 3C).

Figure 3D illustrates the K112 and Y113 residues of the AMP-binding site. These two residues were mutated to alanine to eliminate AMP hydrogen bonding to amino acids in the binding pocket. Notably, the overlay of pig kidney and human not only align, but are also in nearly identical orientation in both species. Additionally, the Y164 and M177 residues were found in close proximity, connected to the active site (Figure 3D).

Finally, Figure 3E shows residue M248 positioned near the triad of acidic residues co-ordinating manganese (Mn; an activating metal), and is found in the active site to co-ordinate F6P. The M248 residue was mutated to aspartic acid in an attempt to activate the enzyme as a means to enhance its binding affinity to the activating metals manganese and magnesium.

### Kinetic analysis of FBPase mutants and comparison with WT enzyme

Initially, IC_50_ of AMP for mutants K112A and Y113A was determined at fixed concentrations of FBP substrate (five increasing concentrations of AMP from 2.5 to 80 µM (Figure 4A and Table 1). The IC_50_ values showed a six- to nine-fold increase for these two mutants relative to the WT enzyme. In contrast, Y164A and M177A mutants demonstrated a two-fold decrease in both AMP IC_50_ and F2,6-BP IC_50_ relative to the WT. Conversely, mutants L56A and L73A exhibited a five-fold increase in IC_50_ for F2,6-BP inhibitor, and mutant M248D displayed a seven-fold increase in IC_50_ for F2,6-BP (Figure 4B and Table 1).

**Figure 4:** Inhibition of FBPase mutants K112, Y113A, Y164, M177A, M248D, L56A, and L73A (**A**) **Inhibitory curve for WT and mutants K112, Y113A, Y164A, and M177A.** Relative SA is shown for each mutant compared with WT in increasing concentrations of the AMP inhibitor. (**B**) **Inhibitory curve for WT and mutants M248D, L56A, and L73A.** Relative SA is shown for each mutant compared with the WT in increasing concentrations of F2,6-BP inhibitor.

The article "Characterization of recombinant fructose-1,6-bisphosphatase gene mutations: evidence of inhibition/activation of FBPase protein by gene mutation" was published in 2019. Journal: Biosci Rep.

A representative inhibitory curve for each mutant in comparison with the WT enzyme is presented in Figure 4. The relative SA of WT and mutants K112A, Y113A, Y164A, and M177A is shown in Figure 4A as a function of increased concentration of AMP inhibitor. Likewise, the relative SA of WT and mutants M248D, L56, and L73 is shown in Figure 4B as a function of increased concentration of F2,6-BP inhibitor. Mutants K112A, Y113A, Y164A, and M177A exhibited higher enzymatic activity with increased concentrations of AMP inhibitor, compared with the WT (Figure 4A), respectively. Figure 4B presents a decrease in the relative SA for each mutant in response to an increase in F2,6-BP inhibitor concentration, confirming mutant inhibition. Note that M248D mutant is not as strongly inhibited by F2,6-BP as the other mutants or WT enzyme.

At last, a kinetic curve is shown for each mutant in comparison with the WT in Figure 5. Velocity (in units of µmoles/min) compared with increased FBP substrate concentration is shown for FBPase mutants L56A, L73A, Y164A, M177A, and M248D in Figure 5A, and for mutants K112A and Y113A in Figure 5B below.

**Figure 5:** Kinetic curve of FBPase mutants L56A, L73A, Y164A, M177A, M248D, K112A, and Y113 in fixed concentrations of FBP (**A**) Velocity compared with FBP substrate concentration curve for determination of apparent *K*_m_ for WT and mutants L56A, L73A, Y164A, M177A, and M248D (see ‘Materials and methods’ section for details of curve fitting). (**B**) Velocity compared with FBP substrate concentration curve for determination of apparent *K*_m_ for WT and mutants K112A, and Y113.

Figure 5A reflects an increase in kinetic activity at higher substrate concentrations for mutants L56, L73, and M248 compared with the WT, with M248 exhibiting the largest increase in activity. However, mutants Y164A and M177A (Figure 5A) showed a relative decrease in kinetic activity compared with the WT. In contrast, both mutants K112A and Y113 (Figure 5B) displayed an elevation in kinetic activity compared with the WT.

As lower *K*_m_ values correspond to a higher binding affinity of the enzyme to the substrate, and higher *K*_m_ values reflect a lower binding affinity of the substrate to the enzyme, obtaining relevant apparent *K*_m_ values for each mutant served as a means to reveal how tightly bound the active site of each mutant was to the FBP substrate (µM). An approximate 50% reduction in *K*_m_ was observed for mutants K112A and Y113A compared with the WT, with apparent *K*_m_ values of 3.25 and 2.50 µM, respectively (Table 2). Based on this information, K112A and Y113A mutants displayed 2× greater binding to the FBP substrate compared with WT (Table 2). M248D showed the highest binding affinity toward the FBP substrate of all mutants tested with an apparent *K*_m_ value of 1.25 µM, nearly 4× smaller than WT (Table 2).

The article "Characterization of recombinant fructose-1,6-bisphosphatase gene mutations: evidence of inhibition/activation of FBPase protein by gene mutation" was published in 2019. Journal: Biosci Rep.

**Table 2:** Kinetic parameters of interfacial mutants and active site mutants of pig kidney FBPase

Enzyme	*V*_max_ (µM/min)	*K*_m_ (µM)	*k*_cat_ (s^−1^)	CE (*k*_cat_/*K*_m_ )	AMP Hill coefficient
Y164A	27.5	5.30 (± 0.6)	13.5 (± 1.2)	2.60	2.8 (± 0.2)
M177A_1	26.1	4.20 (± 0.6)	12.8 (± 1.3)	3.10	2.6 (± 0.2)
M177A_2*	23.4	4.80 (± 0.5)	11.5 (± 1.2)	2.40	2.8 (± 0.1)
K112A	54.7	3.25 (± 0.2)	26.8 (± 2.5)	8.25	1.0 (± 0.1)
Y113A	55.5	2.50 (± 0.3)	27.2 (± 2.6)	10.9	1.2 (± 0.1)
M248D	62.2	1.25 (± 0.4)	30.5 (± 2.9)	24.4	2.5 (± 0.2)
L56A	52.3	5.20 (± 0.2)	25.6 (± 1.9)	4.90	2.3 (± 0.2)
L73A	50.5	5.10 (± 0.3)	22.5 (± 2.8)	4.41	2.1 (± 0.2)
WT	41.8	4.80 (± 0.5)	20.5 (± 1.2)	4.30	2.2 (± 0.1)

* Second clone tested.

Furthermore, the CE—calculated as k_cat_/*K*_m_—of mutants Y164A and M177A reflected a two-fold decrease in kinetic efficiency compared with the WT enzyme, whereas L56A and L73A showed a five-fold increase in CE (Table 2). Mutants K112A and Y113A displayed an approximately two-fold increase in CE compared with the WT, with Hill coefficient values toward AMP of 1.0 and 1.2, respectively (Table 2). Mutant M248D, however, demonstrated the largest increase in activity, exhibiting an approximate six-fold enhancement in kinetic catalytic efficiency (CE) with respect to the WT, with CE values of 24.4 compared with 4.3 (Table 2), respectively.

Apparent *K*_m_ is in units of micromolar amount of substrate FBP. *V*_max_ is calculated from data in units of micromoles inorganic phosphate/min. *K*_cat_ = *V*_max_/[E], where [E] is the concentration of the enzyme in µM.

Table 3 shows M248D with 6× higher *K*_i_ toward F2,6-BP, a natural heterotropic inhibitor of FBPase, compared with WT. In contrast, the *K*_a_ of magnesium for M248D is approximately six-fold lower than the WT. Both Y164A and M177A showed a nearly two-fold decrease in *K*_i_ for F2,6**-**BP compared with WT. L56 and L73 mutants have 5× higher *K*_i_ values toward F2,6-BP than WT enzyme. Interestingly, they both have a slightly elevated Hill coefficient relative to WT enzyme.

**Table 3:** Kinetic data comparison (*K*_i_ and *K*_a_) of WT and pig kidney FBPases mutants for F2,6-BP and magnesium

Enzyme	F-2,6-BP (µM)	Mg^2+^ (mM)	
	*K*_i_	*K*_a_	Hill coefficient
WT	0.25 (± 0.02)	0.50 (± 0.18)	2.10 (± 0.15)
M248D	1.50 (± 0.23)	0.08 (± 0.02)	2.20 (± 0.17)
K112A	0.24 (± 0.02)	0.51 (± 0.15)	1.98 (± 0.15)
Y113A	0.25 (± 0.02)	0.48 (± 0.16)	2.00 (± 0.19)
Y164A	0.15 (± 0.03)	0.50 (± 0.15)	2.15 (± 0.12)
M177A	0.17 (± 0.02)	0.49 (± 0.18)	2.05 (± 0.12)
L56A	1.25 (± 0.03)	0.52(± 0.13)	2.75 (± 0.16)
L73A	1.35 (± 0.04)	0.48 (± 0.17)	2.95 (± 0.17)

DSF assay was run on WT and each mutant in the absence and presence of AMP and Magnesium activating metal. This was done as a way to determine the stability of the enzymes (by melting point) and to verify whether or not the mutants alter AMP and magnesium binding relative to WT enzyme.

The article "Characterization of recombinant fructose-1,6-bisphosphatase gene mutations: evidence of inhibition/activation of FBPase protein by gene mutation" was published in 2019. Journal: Biosci Rep.

The WT enzyme melting point increased slightly in the presence of AMP and decreased moderately in magnesium. M248D melting point was slightly higher than WT and decreased in presence of AMP and increased in presence of magnesium. K112A and K113A exhibited lower melting point that WT that decreased significantly in the presence of AMP but not significantly changed in the presence of magnesium. Y164A and M177A showed melting points close to WT which did not decrease in the presence of AMP or magnesium. Finally, L56A and L73A showed melting point comparable with WT that did not change in the presence of AMP and Magnesium.

## Discussion

The work herein was performed using the pig kidney FBPase construct. When compared with human amino acids, the pig kidney FBPase gene sequence shared nearly identical architecture to the human, with the exception of two amino acids outside the active site (Figure 2) [1,33]. More specifically, the sequence alignment of amino acids for the human and pig kidney supports the classification of nearly identical architecture (Figure 2). The pig kidney enzyme was used in place of the human enzyme due to difficulty in achieving proper solubility levels of the human recombinant FBPase necessary to perform all of the kinetic assays.

The significant increase in AMP IC_50_ for K112A and Y113A mutants (seven to nine-fold increase; Table 1), coupled with lower apparent *K*_m_ and higher CE compared with WT (Table 2) may be due to a possible disruption in the AMP-binding site architecture, which is linked to the active site of the enzyme by means of hydrogen bonding/hydrophobic interaction networks (Figure 3B). Melting point data from Table 4 reflects an approximately 6° decrease in melting temperature when comparing K112A and Y113A mutants with WT. Additionally, there is approximately 5–9° reduction in melting temperature of K112A and Y113A between mutants in the absence of a ligand, and mutants in the presence of AMP (Table 4).

**Table 4:** Comparison of melting points (°C) of WT and mutant pig kidney FBPases for AMP and magnesium

Enzyme	No Ligand	AMP (100 µM)	Mg^2+^ (2.5 mM)
WT	56.0 (± 2.75)	59.0 (± 1.75)	50.0 (± 1.25)
M248D	62.0 (± 1.25)	59.0 (± 2.50)	65.0 (± 1.75)
K112A	51.0 (± 2.50)	42.0 (± 2.50)	51.0 (± 2.50)
Y113A	50.0 (± 2.25)	45.0 (± 1.25)	52.0 (± 1.50)
Y164A	55.4 (± 2.25)	55.0 (± 2.25)	55.2 (± 1.75)
M177A	54.2 (± 1.75)	54.1 (± 1.25)	55.8 (± 1.75)
L56A	56.0 (± 3.00)	57.0 (± 2.75)	56.0 (± 2.50)
L73A	55.8 (± 2.50)	56.0 (± 3.00)	56.5 (±2.25)

Moreover, the allosteric transition from the active R-state to the inactive T-state of the enzyme may be prevented [10,34] in the K112A and Y113A mutants. More specifically, this increase in the AMP IC_50_ for K112A and Y113A indicates AMP sensitivity is dramatically decreased such that the mutant enzyme would remain in an activated state *in vivo*. Additionally, the K112A Hill coefficient for AMP-binding (Table 2) decreased to 1.00, signifying that co-operative binding of AMP is no longer apparent or present for this mutant. The two-fold increase in CE for both K112A and Y113A mutants is curious, as these data may indicate that subtle changes in active site architecture may result from possible disruption of supporting networks of hydrophobic residues and hydrogen-bonded residues connecting the active site to the AMP-binding site [10] (see Table 4 data).

The article "Characterization of recombinant fructose-1,6-bisphosphatase gene mutations: evidence of inhibition/activation of FBPase protein by gene mutation" was published in 2019. Journal: Biosci Rep.

Importantly, these results suggest that if either K112A or Y113A mutations were to occur naturally *in vivo*, or any other mutation which similarly disrupts hydrogen bonding in the AMP-binding site, the production of F6P product would no longer be controlled by AMP, and feedback inhibition would be lost. As a follow-up to previous studies [35], the structure of an AMP site mutant would elucidate architectural differences in the AMP-binding site, and would confirm the occurrence of a disrupted hydrogen bonding network between the active site and AMP-binding site.

The changes in kinetic parameters for the Y164A and M177A mutants were subtle yet compelling. The IC_50_ values (Table 1) were between 40 and 60% of the WT IC_50_, implying that these mutants are slightly more sensitive to AMP than the WT. Moreover, as shown in Table 2, there is a decrease in CE relative to the WT which suggests that these mutants may have an effect on active site residues to which they are connected via hydrogen bonding network(s) in the FBPase structure. Interestingly, in Table 3, the *K*_i_ decreased for F2,6-BP relative to the WT, indicating that these mutants are more sensitive to inhibition by F2,6-BP.

With respect to the position of M248 in the WT enzyme, the active site mutation target in our study (M248D) is shown in close proximity to an activating manganese metal in the crystal structure. This motivated us to change the methionine to aspartic acid to see if, in the presence of magnesium activating metal, the mutant would be more active than the WT.

The article "Characterization of recombinant fructose-1,6-bisphosphatase gene mutations: evidence of inhibition/activation of FBPase protein by gene mutation" was published in 2019. Journal: Biosci Rep.

From the data presented, M248D can be classified as an ‘activated’ mutant. Although the AMP IC_50_ in Table 1 does not differ from the WT, the IC_50_ value for the active site inhibitor F2,6-BP is 7× greater, corresponding to a lower affinity for inhibition. With reference to Table 2, it is noted that the apparent *K*_m_ decreases by nearly four-fold relative to the WT. This implies an occurrence of tighter binding action, and is further supported by an observed six-fold increase in CE, suggesting that the mutant enzyme is more efficient than the WT. These results are consistent with a 6.25 decrease in *K*_a_ for magnesium binding, as seen in Table 3. Furthermore, a crystal structure of the M248D mutant would provide information about architectural changes in the active site as a result of mutation. Evidence for architectural changes can be seen in Table 4 showing an elevated melting point in the absence of ligand as well as subtle decrease in presence of AMP and increase in melting point in presence of magnesium metal.

L56A and L73A mutants were performed with the purpose of disrupting FBPase interactions with allosteric PFE inhibitor. Unfortunately, this inhibitor is not commercially available to be tested. These interfacial mutants from the PFE Allosteric Binding Site approach the active sites. From Table 1 (and Figure 4B) the 5× increase in IC_50_ of F2,6-BP and 5× higher K_i_ (Table 3) indicate that these mutants may affect active site architecture. However, the F2,6-BP was not heat stable enough to measure the melting point of WT and mutant FBPases in the presence of this inhibitor. From Table 2 and Figure 5A, the L56A and L73A show similar *K*_m_ and Hill coefficient to the WT enzyme.

Analysis of the data presented herein indicates that AMP inhibition is compromised when the FBPase enzyme is mutated. Additionally, the mutant enzymes K112A, Y113A, and M248D were clearly ‘activated’ relative to the WT via loss of inhibition, while Y164A and M177A interfacial mutations between the AMP-binding site and the active site were more easily ‘inactivated’ via inhibition relative to WT. Our data support the theory that mutations in the coding region of FBPase may potentially exacerbate hyperglycemia or hypoglycemia (previously reported in the clinical setting) *in vivo* [2].

However, *in vivo*, the complexity of the signaling system regarding the transport of glucose out of the liver may limit the ability of researchers to directly correlate mutant FBPase activity with blood glucose levels. More work needs to be done *in vivo* in correlation to FBPase mutations, enzymatic activity, and the effects these mutations have on blood glucose levels. If active site mutations such as M248D exist in the FBPase gene product (may be confirmed through clinical studies of patients with hyperglycemia), then new regimes for drug treatments for this disorder may be explored as based on previous drug studies [36,37].

The article "Characterization of recombinant fructose-1,6-bisphosphatase gene mutations: evidence of inhibition/activation of FBPase protein by gene mutation" was published in 2019. Journal: Biosci Rep.

Interpretation of kinetic data tells us that a presence of specific mutations in the coding region of this gene may possibly deregulate the enzyme such that the rate of production of F6P increases dramatically, leading to enhanced gluconeogenesis (glucose production) in direct correspondence to activation of the enzyme where AMP inhibition is lost.

## Abbreviations

CE: catalytic efficiency
DSF: differential scanning fluorimetry
FBP: fructose-1,6-bisphosphate
FBPase: fructose-1,6-bisphosphatase
F2,6-BP: fructose-2,6-bisphosphate
F6P: fructose-6-phosphate
*K*_a_: association (binding) constant
***k***_cat_: catalytic constant
*K*_i_: equilibrium inhibitory constant
*K*_m_: Michelis constant
OD: optical density
PFE: {4-[3-(6,7-diethoxy-quinazolin-4-ylamino)-phenyl]-thiazol-2-yl}-methanol
SA: specific activity
*V*_max_: maximum velocity
WT: wild-type
